This article has been retracted.

# Mobile phone text messaging and Telephone follow-up in type 2 diabetic patients for 3 months: a comparative study

**DOI:** 10.1186/2251-6581-11-7

**Published:** 2012-08-24

**Authors:** Mirta Zolfaghari, Seyedeh A Mousavifar, Hamid Haghani

**Affiliations:** 1 Nursing & Midwifery Care Research Center, Tehran University of Medical Science, Tohid Sq. East Nosrat Street, Tehran, Iran; 2 School of Nursing and Midwifery, Tehran University of Medical Science, Tehran, Iran; 3 Department of Biostatistics, Tehran University of Medical Sciences, Tehran, Iran

**Keywords:** Glycosylated hemoglobin, Cellular phone, Short Message Service, Type 2 diabetes mellitus, Telephone follow-up

## Abstract

**Background:**

To investigate and to compare the effectiveness of a nurse short message service (SMS) by cellular phone and telephone follow-up by nurse on Glycosylated hemoglobin (HbA1c) levels in people with type 2 diabetes.

**Methods:**

Semi experimental study consisted of 77 patients with type 2 diabetes that randomly assigned to two groups: telephone follow-up (n = 39) and short message service (n = 38). Telephone interventions were applied by researcher for 3 months. SMS group that received message daily for 12 weeks. Data gathering instrument include data sheet to record HbA1c and questionnaire that consisted of demographic characteristics. Data gathering was performed at two points: initial the study and after 12 weeks. Data analyzed using descriptive and inferential statistics methods with SPSS version 11.5.

**Results:**

Demographic variables were compared and all of them were homogenous. Results of this study showed that both interventions had significant mean changes in HbA1c; for the telephone group (p = 0.001), with a mean change of −0.93% and for the SMS group (p = 0.001), with a mean change of −1.01%.

**Conclusion:**

Finding of this research showed that intervention using SMS via cellular phone and nurse-led-telephone follow up improved HbA1c for three months in type 2 diabetic patients and it can consider as alternative methods for diabetes control.

## Introduction

The prevalence of diabetes has been alarmingly increasing [1]. Each year, 7 million people are diagnosed with the disease, and every 10s, a person dies from diabetes-related causes [1]. Diabetes is a chronic disease requiring lifelong medical and nursing intervention and lifestyle adjustment [2]. The National Survey of Risk Factors for Non-Communicable of Iran, which was conducted in 2005, demonstrated that the prevalence of diabetes mellitus in Iranian citizens aged 25–64 years was 7.7% (2 million individuals) [3], among whom half are undiagnosed [4]. An additional 16.8%, or 4.4 million, of Iranian adults have impaired fasting glucose [4]. If current trends continue, based on the World Health Organization forecast for Iran, there will be 5.2 million Iranians with diabetes mellitus in 2025[3].This high prevalence of diabetes in working aged adults is an ominous sign for this developing nation [4]. As the relatively young Iranian population ages in the future, and urbanization continues or accelerates, the prevalence of diabetes will likely escalate [4].

The Diabetes Control and Complications Trial showed that for every 1% reduction in the HbA1c levels, there was a 40% to 50% reduction in risk for microvascular and neuropathic complications [5,6]. The American Diabetes Association (ADA) has recommended that all persons with diabetes should attempt to achieve near normalization of blood glucose levels [7].

Algorithms for diabetes care exist but may be complex and difficult for physicians to follow, given the patient load, diversity of patient seen, lack of information systems, and time constraints [8]. In addition, economic and technical barriers to providing diabetes care in the community health system are recognized [9].

Since control of diabetes has been shown to decrease mortality and prevent long-term complications, it is critical that healthcare systems develop innovative ways to improve diabetes management, and provide timely care to patients [1]. Several research studies have shown that various telemedicine approaches can have a positive impact on patient blood glucose control and that over the long term; these approaches can result in reduction or elimination of the complication related to diabetes mellitus [10]. Telemedicine has, in particular, caught the attention of patients and caregivers [1]. For patients, it has the advantage of providing a quick, efficient way to communicate with their providers [1]. Especially, for those patients living in rural areas, it is potentially invaluable to have access to their caregiver from the comfort of their homes, thus sparing them the time and cost of traveling [11]. Although the magnitude of the impact of telemedical support on diabetes care remains debatable [11]. Telemedicine cannot replace patient visit and direct interaction with providers, but it can supplement between-visit care and improve ‘quality of care’ [1]. Patient suffering from chronic diseases in general and diabetes in particular, have benefited from support systems and telephone education with improved clinical outcomes [11], a telephone care program has been shown to be a viable strategy for bringing diabetes management services into patients’ homes, improving their glycemic control and provide timely care to patients [8]. To maintain normal range of blood glucose and prevent diabetic complications, patients ought to contact more frequently with their health care providers, but this will in turn increase health care expenditure [12]. And the telephone intervention was more time- consuming than an Internet-based blood glucose monitoring system [13].

Recently mobile phones as a new delivery system can provide medical recommendations and prescriptions at the appropriate time and to accommodate for patients’ behavioral changes and to normalize of blood glucose levels [14]. Mobile phones are an integral part of everyday life, although mobile phone technology is a relatively new and innovative methodology [15]. This method is becoming an important way of encouraging better nurse-patient communication and will undoubtedly increase in application over coming years [15]. Because of widespread usage and ubiquitous availability of mobile phones these devices may be can maximize the efficiency [16] Using short message service enables users to send and receive text messages to and from mobile phones up to 160 characters [16]. SMS allows rapid reception and reply at low cost. It is an interactive service, and is simple, fast and confidential [17]. Although it has been used for patient reminders, psychological support, medical appointments, to report critical medical events or laboratory results and even for surveys in other countries [17], but no research has been done to test the direct effects of Short Message Service on controlling (HbA1c) in people with type 2 diabetes mellitus and in healthcare delivery in Iran as far as we are aware.

The present study evaluated and compared whether an intervention using the short message service (SMS) of cellular phone by a nurse and nurse-led telephone follow up could improve HbA1c levels in patients with type-2 diabetes mellitus.

## Methods

### Participants

This study is quasi experimental research. Participants were recruited from the Iranian Diabetes Association. We studied this intervention during a three month period starting in May 2008. Diabetes was diagnosed according to the American Diabetes Association (ADA) criteria. The age range was 18–65 years. Patients had to have telephone access in their homes and have their own personal mobile phone, or have access to one belonging to a relative. Although selection criteria required that participants should be diabetic patients that only use Oral anti-diabetic medications, should be able to read and write, have power vision sufficient, no problem in hearing and vocalization and no history of psychiatric diseases. Patients were excluded if they had a clinical history of an important illness such as renal insufficiency with a creatinine level >1.5 mg/dl, hepatic insufficiency, were mentally ill or had less than 7% of HbA1c.

Seventy nine patients met the above criteria and agreed to participate. They were randomized by random permuted block design using a random number table and assigned to one of two groups: SMS group (N = 39) or Telephone group (N = 40). Only 77 subjects completed the entire study, 38 SMS and 39 Telephone. Two subjects were lost before completing the post-test in the Telephone group: one decided to opt out of the programme before completing the post-test and one expired during intervention. One subject was lost before completing the post-test in the SMS group because the change of therapeutic regimen from oral anti-diabetic agents to insulin.

Ethics committee approval was required. For ethical considerations, the research protocol was approved by the Medical Research Ethics Committee of the Tehran University of Medical Sciences. Written consent was obtained from those patients who agreed to participate in the study. Anonymity and confidentiality were guaranteed to participants.

### Intervention

The goal of the intervention was to maintain blood glucose levels within a normal range. Participants attended in three days diabetes self-care education in Iranian Diabetes Association. Before the intervention, each patient was instructed, for 10 minutes by researcher, about how to use their own cell phones and to check their ability to read Short Messages and match the time for telephone follow-up. The researcher provided the intervention for 12 weeks. Patients in the SMS group received about 4 messages weekly consisted of diet, exercise, diabetic medication taking and frequent self-monitoring blood glucose levels. Participants in SMS group could receive our messages at any place where access was possible by cellular phone. The researcher sent optimal recommendations back to each patient, 4 times by short message service of cellular phone weekly. For example, recommendations included: ‘Do you know, the best bread for you is pebble bread’; ‘Please eat vegetables and salad in every meal’; ‘Please for prevention of high glycemic fluctuations’, eat your meals in six times instead of three times’; ‘Please consume your drugs on prescribed times’ ; ‘Do you know, eating in regular times, helps you to control your diabetes better’; ‘Lack of exercise may be the cause of the aggravated glucose level’; ‘Try to exercise 3 times daily and at least 15 minutes every time’; ‘Do at least 30 minutes of physical exercise or walking’; ‘Please check the amount that you eat’; ‘Take your recommended diabetic medication’; ‘If you consume Glybenclamide, please eat it, 30 minutes before your meal’ and so on. The 12 weeks of intervention consisted of continuous education and reinforcement of diet, exercise, medication taking, as well as frequent self-monitoring of blood glucose levels.

The intervention for Telephone group was provided via telephone for 12 weeks. The 12 weeks of intervention consisted of counseling on the nature of the disease, risk factors, importance of maintaining blood glucose levels within a near-normal range, continuous education and reinforcement of diet, exercise, medications taking, hypoglycemia management, illness management how to record daily blood glucose and frequent self-monitoring of blood glucose levels. The researcher contacted the telephone group at least twice a week for the first month and then weekly for the second and third month. The total frequency of telephone counseling averaged 16 times per subject. The duration of each counseling session was an average of 20 minutes. The researcher was asking questions such as: “did you take your recommended diabetic medication?” “When did you consume your prescribed tablet?” Do you know how you’re consuming medications, act in your body? “How many times did you do physical exercise or walking during last days?” “When is the best time to do exercise?” “Did you feel better after doing exercise?” Do you know that doing exercise is as important as diabetic medication?“ How many days did you follow your recommended diet over the past days?” Did you eat salad and vegetable before every meal?” Before initiation of recommendation, researcher asked every patient about problems they were facing during last days and patients could ask their questions and could solve their problems. Sometimes they feel stress, so the researcher educate some ways of decreasing stress such as: deep breathing, distraction methods, taking a bath, go to the country, concentrate to good points of their life, be more with their family members or closed or lovely friends, try to laugh more and so on.

### Procedure

Before the intervention, demographic characteristics and HbA1c value were collected as pre-test data at the Iranian Diabetes Society. The intervention was provided to the telephone group with counseling appointments scheduled when convenient to the subject. The HbA1c was measured again three months later. Patients’ blood was drawn in veins for HbA1c measurement. HbA1c was measured in the metabolism and endocrinology laboratory of the Tehran University-affiliated medical center. HbA1c was determined by a high-performance liquid chromatography technique. HbA1c level was measured after 12 weeks as posttest data.

### Data analysis

The data were analyzed using the SPSS (Version 11.5) program. Chi square test, Paired t-test, independent t-test and Fisher’s exact test were used to test for the homogeneity of demographic and clinical characteristics between the SMS and Telephone groups. The paired t test was used for comparison of differences between pretest and posttest values in the group. The unpaired t test was used for comparing the differences between the SMS and Telephone groups.

## Results

The characteristics of the SMS and Telephone groups are shown in Table 1. The mean age of the SMS group was 51.07 years and that of Telephone group was 53.71 years. The mean BMI of the SMS group was 29.008 kg/m^2^ and that of Telephone group was 27.334 kg/m^2^. There was no significant difference in age, gender, BMI, duration of diabetes, treatment method and blood glucose levels between the two groups.

**Table 1:** Baseline demographic and clinical data of the SMS and intervention groups

**Characteristics**	**SMS group (n = 38)**	**Telephone group (n = 39)**	**t / χ^2^**	**p**
Age (years)	51.70 ± 9.90	53.71 ± 9.04	1.221	0.226
Sex:Male/.Female	18/20	18/21	0.011	0.915
Body mass index (kg.m^2^)	29.008 ± 6.65	27.334 ± 3.53	1.374	0.175
Diabetes duration (months)	95.57 ± 72.96	74.55 ± 61.93	1.365	0.176
Glycosylated haemoglobin (%)	8.97 ± 1.65	9.44 ± 1.72	1.219	0.227

Data are Means ± SD (%).

At the pre-test, no significant differences were found in HbA1c between the groups in Table 1. HbA1c did not differ significantly with two groups (SMS group vs. Telephone group) (p = 0.227). There was a significant percentage change in HbA1c for the SMS group (p = 0.000), with a mean change of −1.01 (8.97% pre-test to 7.96% three months), and also there was a significant percentage change in HbA1c for the Telephone group (p = 0.000), with a mean change of −0.93 (9.44% pre-test to 8.51% three months).

Glycosylated hemoglobin (HbA1c) decreased 0.93% points at three months compared with baseline in the Telephone group and 1.01% points at three months compared with baseline in the SMS group (Table 2). There was no significant difference were found between two intervention (p = 0.186).

**Table 2:** Effect of the intervention on Glycosylated haemoglobin (%) levels

**Variable HbA_1_C (%)**	**Baseline**	**3 months**	**Difference (Post-test) – (Pre-test)**	**t**	**p**
SMS group	8.97 ± 1.65	7.96 ± 1.75	−1.01 ± 0.01	4.254	0.000
Telephone group	9.44 ± 1.72	8.51 ± 1.85	−0.93 ± 0.13	4.150	0.000

## Discussion

Glycosylated haemoglobin reflects mean blood glucose levels over the previous six weeks. HbA1c has become a standard assessment of glycaemia and a standard part of diabetes management [7]. Therefore, large studies of this relationship, such as the Diabetes Control and Complications Trial Research Group (1993) and the United Kingdom Prospective Diabetes Study Group (UKPDS, 1998), used HbA1c as the primary index of glycaemia [5,6].

This study evaluates and compares whether an intervention using the short message service (SMS) of cellular phone by a nurse and nurse led telephone follow-up would improve HbA1c levels in patients with type-2 diabetes mellitus for three months.

In this study, HbA1c levels decreased 1.01% points in SMS group and 0.93% points in Telephone group after 12 weeks compared with baseline. Previous studies showed the following results: Kwon et al. (2004) reported that the 12-weeks follow-up examination HbA1c levels in diabetic patients by web-based management system using short message service (SMS) caused to mean decrease of 0.9% points in HbA1c [12], People with diabetes in a nurse short-message service by cellular phone intervention group had mean decrease of 1.15% points in HbA1c levels during the 3-months study period and 1.05% points at six months [14]. A short message service by cellular phone study in type 2 diabetic patients resulted in a decrease of HbA1c of 1.31% points at nine months and 1.32% points at twelve months [18]. An SMS intervention study by a nurse showed that the HbA1c levels decreased 1.1 percentage points after 12 weeks [2]. At the end of Internet diabetic patient management study using a Short Messaging Service A1C levels were significantly (0.72%) decreased in the intervention group [19]. The study of evaluating the impact of nurse’s education by short message service of cellular phone and wire internet revealed a significant percentage change in a baseline HbA1c ≥7.0% for the intervention group with a mean change of −2.15(9.35% pretest to 7.20% post-test) at 3-months follow-up [13]. An intervention using SMS of personal cellular phone and internet showed great efficacy in HbA1c control in obese type 2 diabetes. The intervention group showed a marked decrease in HbA1c levels after 12 months of follow-up versus the baseline levels (a mean percentage change of −1.22 at 3 months, -1.09 at 6 months, -1.47 at 9 months and −1.49 at 12 months [20]. Kim, Oh and Lee (2005) reported that a nurse-coordinated intervention by telephone decreased HbA1c levels 1.2 percentage points after 12 weeks [8]. In a prior randomized trial, the effect of nurse telephone calls on HbA1c levels was evaluated. After 12 weeks, patients in the telephone intervention group had a mean decrease of 1.2% in HbA1c levels [21]. These results confirm that the use of various telemedicine approaches can have a positive impact on patients’ HbA1c control.

Therefore, mean end-point HbA1c levels in the intervention groups of the 2 studies were essentially the same. However, in the telephone intervention group, nurse spent more time and money with patients than the SMS intervention by nurse. Overall, the findings suggested that the SMS intervention as improved HbA1c level as telephone group. Patients with diabetes wanted more frequent contact with their health care providers for managing the disease. By using telemedicine management systems such as short message service via cellular phones and telephone follow-up, patients can contact their nurses frequently. The patients in the Telephone group have more frequent contact with the nurse than those in the short message service of cellular phone group. In addition, the patients in the Telephone group received advice according their most recent data, confirming their current state. These factors may have stimulated and motivated the patients to control glucose levels enthusiastically.

These results have important clinical implications because the service for diabetic patients provided via mobile phone is now increasing, whereas the efficacy of the short message service for glucose control has not been evaluated extensively. Also, this study results show evidence that short message services are as effective as telephone calls guidance in managing diabetes. One major advantage of short message service is that the researcher could send short messages without location limitations. An intervention that involves the use of SMS and personal cellular phone can also be applicable to other chronic diseases such as hypertension, hyperlipidemia, obesity, and metabolic syndrome.

This study adds that a nurse educational intervention programme using the telephone calls and an SMS by cellular phone improved levels of glycosylated haemoglobin levels for three months in patients with type2 diabetes. The SMS by cellular phone can be used as a means of providing education for patients with diabetes.

The trial demonstrated the usability of the system. The effectiveness of the system relied on regular contact. The contact frequency provided an indication of the level of acceptance and the extent to which use of the system had become a habit. Therefore, nurse’s education using SMS of cellular phone not only allowed for the patients to maintain steady levels of HbA1c, but also improved the degree of their HbA1c control as well. These results confirm that the use of various telemedicine approaches by the nurse have a positive impact on patient’s HbA1c control.

Although this study demonstrated that an SMS of cellular phone intervention by a nurse could maintain and reduce .HbA1c during a short-term study period of 12 weeks, the long-term effectiveness remains to be determined.

In this study, Iranian patients with type 2 diabetes who received short massages and followed by telephone had improved HbA1c levels. This study suggests both telephone follow-up intervention and using SMS of personal cellular phone improved HbA1c levels remarkably during three months in type 2 diabetic patients. Regard to convenience of SMS can be used as an appropriate alternative method for following up in diabetic patients.

## Competing interests

The authors declare that they have no competing interests.

## Authors’ contributions

MZ had substantial contributions to conception and design of the study, analysis of the data and drafting the manuscript. SAM had substantial contributions to acquisition of data and analysis. HH involved in the data analysis and the interpretation of results. All authors read and approved the final manuscript.

## References

[B1] AzarMGabbayRWeb-based management of diabetes through glucose uploads: Has the time come for telemedicine?diabetes research and clinical practice20098391710.1016/j.diabres.2008.09.05519056140

[B2] KimHSKimNCAhnSHImpact of a nurse short message service intervention for patients with diabetesJournal of nursing care quality20062126610.1097/00001786-200607000-0001216816608

[B3] AminiMParvareshEPrevalence of macro-and microvascular complications among patients with type 2 diabetes in Iran: a systematic reviewdiabetes research and clinical practice200983182510.1016/j.diabres.2008.10.01019091437

[B4] EsteghamatiAMeysamieAKhalilzadehORashidiAHaghazaliMAsgariFKamgarMGouyaMAbbasiMThird national Surveillance of Risk Factors of Non-Communicable Diseases (SuRFNCD-2007) in Iran: methods and results on prevalence of diabetes, hypertension, obesity, central obesity, and dyslipidemiaBMC Publ Health2009916710.1186/1471-2458-9-167PMC269798919480675

[B5] TurnerRHolmanRCullCStrattonIMatthewsDFrighiVManleySNeilAMcelroyKWrightDIntensive blood-glucose control with sulphonylureas or insulin compared with conventional treatment and risk of complications in patients with type 2 diabetes (UKPDS 33)Lancet19983528378539742976

[B6] ReichardPNilssonBYRosenqvistUThe effect of long-term intensified insulin treatment on the development of microvascular complications of diabetes mellitusN Engl J Med199332930430910.1056/NEJM1993072932905028147960

[B7] AssociationADStandards of Medical Care for Patients With Diabetes MellitusDiabetes Care199720S3S13

[B8] KimHSOhJALeeHOEffects of nurse-coordinated intervention on patients with type 2 diabetes in KoreaJournal of nursing care quality20052015410.1097/00001786-200504000-0001115839295

[B9] ZgiborJCSongerTJExternal barriers to diabetes care: addressing personal and health systems issuesDiabetes spectrum200114232810.2337/diaspect.14.1.23

[B10] MeaseAWhitlockWBrownAMooreKPavliscsakHDingbaumALacefieldDBukerKXenakisSTelemedicine improved diabetic managementMilitary Medicine200016557910957848

[B11] JacksonCLBolenSBrancatiFLBatts-TurnerMLGaryTLA Systematic Review of Interactive Computer‐assisted Technology in Diabetes CareJournal of general internal medicine2006211051101639051210.1111/j.1525-1497.2005.00310.xPMC1484664

[B12] KwonHSChoJHKimHSLeeJHSongBROhJAHanJHChaBYLeeKWDevelopment of web-based diabetic patient management system using short message service (SMS)diabetes research and clinical practice200466S133S1371556396410.1016/j.diabres.2003.10.028

[B13] Hee-SungKImpact of web‐based nurse’s education on glycosylated haemoglobin in type 2 diabetic patientsJ Clin Nurs2007161361136610.1111/j.1365-2702.2007.01506.x17584355

[B14] KimH-SJeongH-SA nurse short message service by cellular phone in type-2 diabetic patients for six monthsJ Clin Nurs2007161082108710.1111/j.1365-2702.2007.01698.x17518883

[B15] BlakeHInnovation in practice: mobile phone technology in patient careBritish Journal of Community Nursing2008131601651859530310.12968/bjcn.2008.13.4.29024

[B16] KollmannAHaynDKastnerPSchreierGMobile phones as user interface in the management of chronic diseasese & i Elektrotechnik und Informationstechnik200612312112310.1007/s00502-006-0327

[B17] Ferrer-RocaOCardenasADiaz-CardamaAPulidoPMobile phone text messaging in the management of diabetesJournal of telemedicine and telecare20041028228510.1258/135763304202634115494086

[B18] YoonKHKimHSA short message service by cellular phone in type 2 diabetic patients for 12 monthsdiabetes research and clinical practice20087925626110.1016/j.diabres.2007.09.00717988756

[B19] KimCKimHNamJChoMParkJKangEAhnCChaBLeeELimSInternet diabetic patient management using a short messaging service automatically produced by a knowledge matrix systemDiabetes Care2007302857285810.2337/dc06-246417682122

[B20] KimSIKimHSEffectiveness of mobile and internet intervention in patients with obese type 2 diabetesInternational journal of medical informatics20087739940410.1016/j.ijmedinf.2007.07.00617881285

[B21] KimHSOhJAAdherence to diabetes control recommendations: impact of nurse telephone callsJ Adv Nurs20034425626110.1046/j.1365-2648.2003.02800.x14641395

